The article "Astragalus Polysaccharides Promote Wound Healing in Diabetic Rats by Upregulating PETN and Inhibiting the mTOR Pathway" was retracted in 2023. Reasons: signs of a paper mill; compromised peer review; unreliable results or conclusions.

# Astragalus Polysaccharides Promote Wound Healing in Diabetic Rats by Upregulating PETN and Inhibiting the mTOR Pathway

**DOI:** 10.1155/2022/3459102

**Published:** 2022-10-14

**Authors:** Le Ma

**Affiliations:** Department of Dermatology, The First Hospital of Hunan University of Chinese Medicine, Changsha, Hunan 410007, China

## Abstract

**Objective:**

Presently, astragalus polysaccharide (APS) is being investigated for its therapeutic potential in various diseases; however, its underlying mechanism has not yet been clarified. This study was aimed at observing the effects of APS on wound healing in diabetic rats and at exploring its underlying mechanism.

**Methods:**

Streptozotocin was injected into the tail vein of SD rats to induce diabetic animal models, in which an incision on the back was made. Rats were treated with different dosages of APS to observe their wound healing. Additionally, RT-qPCR and Western blot assay were conducted to observe the expression levels of PTEN and mTOR pathway-associated factors.

**Results:**

Diabetic rats had a prolonged wound healing process, fewer blood vessels, and increased inflammatory response, in which decreased PTEN and elevated mTOR phosphorylation were also identified. APS effectively improved wound healing in a dose-dependent manner by inhibiting the release of inflammatory mediators and attenuating endothelial injuries. Suppression of PTEN could effectively increase the phosphorylation of mTOR and diminish the therapeutic functions of APS on wound healing in diabetic rats.

**Conclusion:**

This study highlighted that APS could promote wound healing in diabetic rats by upregulating PTEN and suppressing the mTOR pathway activation.

## 1. Introduction

As a major complication of diabetes, difficulties in wound healing have complicated and multifactorial pathophysiology, which involves vascular, neuronal, biochemical, and immunological components [1]. Wound healing is a dynamic biological process involving several coordinated and overlapping phases, including proliferation, maturation, and coagulation-inflammation [2, 3]. The traditional treatment for diabetic wound healing is to strictly control blood glucose and implement anti-infection strategies. Nevertheless, for those with severe ulcers, this treatment approach has been far from satisfactory [4], urging the need for more effective therapeutics to treat diabetic wounds.

Astragalus polysaccharide (APS) is the most significant natural active ingredient in *Astragalus membranaceus* and was shown to possess multiple pharmacological effects, including low toxicity, nonresidue, nontolerance, and few adverse events [5]. Emerging evidence shows that APS can reduce blood glucose and lipid and induce insulin resistance in diabetic rats [6–8]. In addition, APS has also been reported to relieve diabetic complications. For instance, Yue et al. stated that in high-glucose-induced hepatocytes and rats with type 2 diabetes mellitus, APS alleviated liver endoplasmic reticulum stress [9]. Zhang et al. reported that APS attenuated early diabetic nephropathy [10], regulated glucose and lipid metabolism, and diminished cardiac fibrosis in diabetic cardiomyopathy [11, 12]. Yang et al. found that APS had promising efficacies in treating diabetic skin wounds [4]. Thus, existing literature indicates that APS might be important in regulating wound healing in diabetes. However, the molecular mechanisms of APS in regulating diabetic skin wounds remain unclear.

The article "Astragalus Polysaccharides Promote Wound Healing in Diabetic Rats by Upregulating PETN and Inhibiting the mTOR Pathway" was retracted in 2023. Reasons: signs of a paper mill; compromised peer review; unreliable results or conclusions.

Phosphatase and tensin homolog (PTEN) is differentially expressed in patients with diabetes, and downregulated PTEN was shown to delay wound healing in patients with diabetic foot ulcers [13]. A recent study indicated that PTEN could suppress the phosphorylation of the mammalian target of rapamycin (mTOR), thereby intensifying autophagy and apoptosis of endothelial cells under high-glucose conditions [14]. In this regard, we speculated that APS might affect PTEN expression and the mTOR pathway in diabetic rats.

To improve current understanding and explore the possible mechanism of APS on diabetic wound healing, this study was aimed at observing the effects of different dosage of APS on wound healing in diabetic rats and at investigating the implication of PTEN/mTOR in wound healing.

## 2. Materials and Methods

### 2.1. Ethical Statement

The study protocol was approved by the Animal Ethics Committee of the First Hospital of Hunan University of Chinese Medicine (Hunan, China), and the experimental procedures were performed following the ethical requirements of animal experiments animal ethics No. ZYFY20200210-23.

### 2.2. Experimental Animals

A total of 40 clean-grade male Sprague-Dawley (SD) rats (10-week-old, weighing 290-310 g) were obtained from Shanghai Laboratory Animal Company (SLAC, Shanghai, China). The rats were fed in a specific pathogen-free animal room of the animal center of the First Hospital of Hunan University of Chinese Medicine under the following conditions, maintained at a temperature of 23.0 ± 2.0°C, relative humidity of 40%-60%, and 12-hour day/night cycle. They were given free access to food and water.

### 2.3. Establishment of Diabetic Rat Model, Skin Wound, and Grouping

#### 2.3.1. Establishment of the Diabetic Model

Briefly, the rats were allowed to acclimate to the environment for seven days, then fasted for 12 hours before model establishment. According to a random number table, 5 rats were selected into the control group and were injected with an equal volume of 0.1 mol/L citric acid-sodium citrate buffer via the tail vein. The remaining 35 rats were injected with streptozotocin (STZ) solution (Sigma, St Louis, MO, USA) diluted by 0.1 mol/L citric acid-sodium citrate at a dose of 45 mg/kg once through the tail vein to establish diabetic rat models. Seven days after STZ injection, the caudal venous blood of the STZ-induced rats was collected, and their blood glucose level was assessed. A blood glucose level > 16.7 mmol/L was defined as successful establishment of diabetes models.

The article "Astragalus Polysaccharides Promote Wound Healing in Diabetic Rats by Upregulating PETN and Inhibiting the mTOR Pathway" was retracted in 2023. Reasons: signs of a paper mill; compromised peer review; unreliable results or conclusions.

#### 2.3.2. Establishment of Skin Wound Model

The diabetic rats and rats in the control group were anesthetized via intraperitoneal injection with 30 g/L pentobarbital sodium at a dose of 30 mg/kg. After disinfection with 2% iodophor, a square skin incision with a depth of 1.5 cm × 1.5 cm to the superficial fascia was made at symmetrical parts on both sides of the rats' spine. Immediately after injury, 0.3 mL phosphate-buffered saline (PBS) was evenly applied to the wound surface, and the rats were then housed in separate cages.

#### 2.3.3. Animal Grouping

1. Rats with normal blood glucose not injected with STZ were labeled as the control group. The diabetic rats were divided into the model group, low-dose astragalus polysaccharide (APS) group (APS-L), medium-dose APS group (APS-M), and high-dose APS (APS-H) groups as per the random number table (5 rats in each group). Rats in the APS-L, APS-M, and APS-H groups were given 50, 100, or 200 mg/kg APS (purity > 98%, Lanzhou Wotelaisi Biological Co. Ltd., Lanzhou, China) once a day. Rats in the control and the model groups were intragastrically given the same amount of saline for 2 weeks
2. si-PTEN and si-NC were provided by GenePharma (China), and their sequences were as follows: si-PTEN: 5′-GAC AGC CAT CAT CAA AGA GAT-3′; si-NC: 5′-UUC UCC GAA CGU GUC ACG UTT-3′. si-PTEN as well as its negative control si-NC lentivirus was locally injected into the base and wound margin of the wound in rats. Four injection points were injected into each wound, and 25 *μ*L lentivirus was injected into each of the four upper, lower, left, and right directions of the wound. STZ-induced rats were injected with siRNA-NC and labeled as the model+siRNA-NC group. Local injection of lentivirus knocked down siRNA-PTEN vector to decrease PTEN expression in rats. The diabetic rats were divided into the APS+siRNA-NC and the APS+siRNA-PTEN groups as per the random number table (5 rats in each group)

After the intragastric administration of 200 mg/kg APS, rats' fur was removed after anesthesia with pentobarbital sodium, and a cutaneous skin wound (full thickness, 10 mm in diameter) was made with the application of a punch biopsy needle. Next, the rats were subcutaneously injected with APS around the wounds at 4 different injection sites on the 0, 3^rd^, 7^th^, and 14^th^ day after wounding (25 *μ*L per site).

The article "Astragalus Polysaccharides Promote Wound Healing in Diabetic Rats by Upregulating PETN and Inhibiting the mTOR Pathway" was retracted in 2023. Reasons: signs of a paper mill; compromised peer review; unreliable results or conclusions.

### 2.4. Sample Collection and Treatment

On the 3^rd^, 7^th^, and 14^th^ days of wound establishment, the rats were sacrificed using excessive anesthesia. The back-wound tissues were taken, and a part of which was fixed in 4% neutral formalin solution for the paraffin-embedded sections. The other part was placed in a sterile cell cryopreservation tube, quickly frozen in liquid nitrogen, and then transferred to a -80°C refrigerator for quantitative polymerase chain reaction (qPCR) and Western blot assay. On the 14^th^ day of APS injection, the rats were anesthetized and blood from their common carotid artery was collected. The blood was centrifuged at 3500 r/min for 10 minutes to obtain the serum for examination.

### 2.5. Morphological Observation of the Skin Wound

A scale was placed as a standard after skin wound in rats, which was placed on the edge of the rats' wound and photographed using a digital camera. The ImageJ software was used to calculate the wound healing rate by measuring the unhealed skin wound area: (original wound area − unhealed wound area)/original wound area × 100%. Under aseptic conditions, 5 mm of tissues covering the entire skin wound surface was cut from the wound edge. Then, the tissues were fixed with 4% paraformaldehyde for 48 hours and gradually dehydrated by ethanol, permeabilized by xylene, embedded in the paraffin wax, and sliced continuously using a semiautomatic microtome at a thickness of 4 *μ*m. The sections were taken for hematoxylin and eosin (H&E) staining and Masson staining, and the morphological changes of the wound tissues were captured under an optical microscope (200x magnification).

### 2.6. Immunohistochemistry and Quantitation of Microvessel Density (MVD)

The slices were baked in an oven at 60°C for 1 hour, then dewaxed with xylene, dehydrated with ethanol, and finally washed in ddH_2_O. Next, the slices were boiled in 0.01 M citrate buffer (pH = 6.0), maintained for 10 minutes for antigen retrieval, and incubated with 3% H_2_O_2_ for 10 minutes in the dark to suppress the endogenous peroxidase. Subsequently, the slices were cultured overnight at 4°C with diluted rabbit anti-CD31 primary antibody (dilution: 1 : 200, ab28364) (Abcam, Cambridge, UK), followed by incubation with a secondary antibody for 30 minutes at 37°C. After dripping diaminobenzidine chromogenic solution for color development, the slices were counterstained with hematoxylin, differentiated with 0.5% hydrochloric acid alcohol, followed by gradient alcohol dehydration, xylene clearance, and neutral gum blocking, and the positive reaction was viewed under a light microscope. Brownish-yellow in the cell membrane or cytoplasm was considered as positive expression.

The article "Astragalus Polysaccharides Promote Wound Healing in Diabetic Rats by Upregulating PETN and Inhibiting the mTOR Pathway" was retracted in 2023. Reasons: signs of a paper mill; compromised peer review; unreliable results or conclusions.

Each slice was selected with three regions that showed the most neovascularization characters under 5x magnifications. Then, three areas in each selected region were randomly observed under a magnification of 20x and analyzed using the Image-Pro Plus software. The microvessel density (MVD) was calculated by counting the mean blood vessel per image.

### 2.7. Enzyme-Linked Immunosorbent Assay (ELISA)

By applying the nitric acid reductase method, the absorbance (*A*) value in serum was measured at 550 nm to calculate the concentration of nitric oxide (NO) as per the kit instructions, and the concentration of nitric oxide synthase (NOS) was calculated according to the kit instructions at 530 nm. The ELISA method was implemented for measuring the serum levels of endothelin-1 (ET-1), intercellular adhesion molecule (ICAM-1), interleukin-6 (IL-6), and tumor necrosis factor-*α* (TNF-*α*) as per the kit instructions. The NO and NOS kits were purchased from Nanjing Jiancheng Institute of Biological Engineering (Nanjing, China), IL-6 and TNF-*α* kits from Neobioscience Technology Company (Shenzhen, China), and ET-1 and ICAM-1 kits from ColorfulGene Biological Technology Co., Ltd. (Wuhan, China). Five biological replicates were set, and three duplicate wells were set for each sample.

### 2.8. Reverse Transcription qPCR (RT-qPCR)

The total RNA of real-time PCR was isolated from the rats' wound tissues with the application of TRIZOL, following the manufacturer's requirements. The reverse transcription of RNA to complementary DNA was implemented using the FastQuant RT kit, and the SYBR Green was utilized for the real-time PCR analysis. The primer sequences were as follows: PTEN, forward, 5′-TTTGAAGACCATAACCCACCAC-3′; reverse, 5′-ATTACACCAGTTCGTCCCTTTC-3′; *β*-actin, 5′-CTCCCCCATGCCATCCTGCGTCTG-3′; reverse, 5′-CTCGGCCGTGGTGGTGAAGC-3′. All experiments were performed in triplicate. The target gene mRNA quantification was calculated using the 2^-△△Ct^ method, with *β*-actin as a loading control. Five biological replicates were set, and three duplicate wells were set for each sample.

### 2.9. Western Blot Assay

The cryopreserved wound tissues were ground with liquid nitrogen and added into an EP tube. Next, the tissues were fully lysed, the tissue lysate was used to extract the total protein, and an ultraviolet spectrophotometer was adopted to measure the total protein concentration, followed by plotting the standard curve of the protein concentration. The extracted protein was boiled, denatured, and stored at -80°C for later use. A sodium dodecyl sulfate-polyacrylamide gel electrophoresis was made, to which an equal volume of protein was injected for electrophoresis, transmembrane, and blocking, then probed with the primary antibody against PTEN (dilution: 1: 2000, ab32199), mTOR (dilution: 1: 2000, ab2732), phosphorylated (p)-mTOR (dilution: 1: 1000, ab109268), or *β*-actin (dilution: 1: 1000, ab8277) overnight at 4°C. Afterward, the membrane was reprobed with the secondary antibody for 60 minutes at room temperature, followed by rinsing and development. Lastly, the ImageJ software was processed to detect the gray value of protein bands. Five biological replicates were set.

The article "Astragalus Polysaccharides Promote Wound Healing in Diabetic Rats by Upregulating PETN and Inhibiting the mTOR Pathway" was retracted in 2023. Reasons: signs of a paper mill; compromised peer review; unreliable results or conclusions.

### 2.10. Statistical Analysis

The experimental data are expressed as mean ± standard deviation. The two groups were compared using the independent sample *t*-test, and the multiple groups were compared using the one-way analysis of variance (ANOVA) with Tukey's post hoc test. Statistical analyses were performed using Graph prism 8.0. *P* value less than 0.05 was used as the significance threshold.

## 3. Results

### 3.1. General Conditions of the Rats

#### 3.1.1. Overall Conditions

The rats were classified into a model group, APS-L, APS-M, and APS-H groups. Those in the control group were generally in good condition with shiny fur, normal diet habits, and active and quick response. The diabetic rats were generally in poor condition as they had poor appetite and slowed responses. The conditions of diabetic rats treated with three doses of APS were generally better than those without APS treatment.

#### 3.1.2. Body Weight Changes

No change was observed in the body weight of rats in each group before modeling. After 3, 7, and 14 days since the diabetes modeling, the body weight of each rat was increased. Seven days after the skin wound modeling, the body weight was elevated in rats treated with medium and high dose of APS. On the 14^th^ day after skin wound modeling, the rats treated with medium and high dose of APS had heavier body weights. These results suggested that APS may attenuate diabetes-induced weight loss (Figure 1(a)).

#### 3.1.3. Changes in Blood Glucose

After modeling, the blood glucose of diabetic rats and those treated with three doses of APS was elevated. Fourteen days after modeling, no change was found in blood glucose between diabetic rats and diabetic rats treated with low-dose of APS, while the glucose of rats in the high APS dose group was decreased compared with the other diabetic rats. These results suggested that high dose of APS could decrease the glucose level of diabetic rats (Figure 1(b)).

The article "Astragalus Polysaccharides Promote Wound Healing in Diabetic Rats by Upregulating PETN and Inhibiting the mTOR Pathway" was retracted in 2023. Reasons: signs of a paper mill; compromised peer review; unreliable results or conclusions.

### 3.2. Wound Healing of Rats

On the 3^rd^ day after the skin wound, the wounds of rats in the control group shrank to a smaller area, but the wounds of the other groups did not shrink remarkably. On the 7^th^ day after the skin wound, the wound granulation tissues of rats in the control group had covered the wound and showed a bright red color. It could be seen that the neoepidermis crawled from the periphery to the center of the wound. The wound granulation tissues of diabetic rats were shallow, the wound margin was still deep, and the epidermal repair was not obvious. Similar to the diabetic rats, the rats in the low-dose APS group had shallow wound granulation tissues and unobvious epidermal repair. The growth of the wound granulation tissues of rats was vigorous upon treatment with medium and high dose of APS, and the wound healing was the best in the high-dose treatment. On the 14^th^ day, the neoepidermis of the wound of rats from the control group was matured and thickened, and the color of the wound gradually changed from pink to white. The wound in diabetic rats and rats treated with low-dose APS was still bright red, the epidermis was not obviously repaired, and the wound contraction was not obvious. In rats that received high-dose APS treatment, their wounds were mostly closed, shrank well, and pink. The wounds of the rats with medium-dose APS treatment still had a small number of open wounds, which were covered with bright red granulation (Figure 1(c)).

The wound healing of rats after STZ treatment was slowed down compared with rats in the control group at all time points. The wound healing rate of the open wound was enhanced in diabetic rats on day 14. Low-dose APS had no effects on the wound healing of diabetic rats. Medium- and high-dose APS could promote wound healing in diabetic rats, and the healing rate of these two groups was higher than those of diabetic rats at all time points. Among them, rats with high-dose APS treatment showed the best effect and continued till the end of the observation period (Figure 1(d)).

### 3.3. Morphological Observation of the Wound Tissues of Rats in Each Group

Based on the H&E staining findings of the granulation tissues of the wounds, rats in the control group had thick granulation tissues with constant and complete epidermis structure, along with fibroblast proliferation, while the granulation tissues in the model group were thin with incomplete epidermis structure, in which a small amount of disordered collagenous fibers was observed. The granulation tissues were thicker in the APS-L group, with a more complete epidermis structure and increased fibroblast proliferation and collagenous fibers (Figure 2(a)).

The article "Astragalus Polysaccharides Promote Wound Healing in Diabetic Rats by Upregulating PETN and Inhibiting the mTOR Pathway" was retracted in 2023. Reasons: signs of a paper mill; compromised peer review; unreliable results or conclusions.

Masson staining was used to stain the collagen fibers into blue, which was used to evaluate the deposition of the matrix. Masson staining results showed that 14 days after the skin wound, the rats in the control group had deep blue coloration, and the collagen fibers on the granulation tissues were neatly arranged. The blue coloration in the diabetic rats and rats treated with low-dose APS was the lightest, and the collagen arrangement was sparse and disorderly. The rats treated with medium-dose APS exhibited elevated blue staining and neatly arranged collagen. The rats treated with high-dose APS had improved matrix deposition on the wound, which had the most collagen fibers (Figure 2(b)).

Ki67 staining demonstrated that 14 days after the skin injury, the expression of Ki67 in the model group was decreased compared with that in the control group, while the expression of Ki67 in the APS-H group was substantially elevated compared with that in the model group (Figure 2(c)).

### 3.4. Angiogenesis in Wounds of Rats in Each Group

Angiogenesis is a complex process in which new capillaries sprout from adult blood vessels. To assess wound angiogenesis, we used CD31, a specific marker of vascular endothelial cells, to assess the density of new microvessels in wounds. CD31 immunohistochemical staining results showed that 14 days after the skin wound, the rats in the control group had more microvessels in the wound area. The MVD was decreased in the diabetic rats, which was not significantly different from the rats treated with low-dose APS. MVD was elevated in rats treated with medium-dose APS, which was further elevated in the high-dose APS group. These results show that APS could promote the formation of new blood vessels in the diabetic wound tissue and accelerate the wound healing process (Figures 2(d) and 2(e)).

### 3.5. Expression of Vascular Endothelial-Related Factors and Inflammatory Factors in Rats

Vascular endothelial cells secrete ET-1 and NO to regulate blood vessels' contraction and relaxation. Hyperglycemia and high insulin levels were shown to damage endothelial cells, resulting in an imbalance of ET-1 and NO/NOS, dysfunction of vasoconstriction and relaxation, and aggravation of vascular endometrial damage. In addition, injury of the vascular intima is the basis of vascular disease, which is an important factor associated with diabetic skin ulcers [15, 16]. A high expression of ICAM-1 in vascular endothelial cells may further promote the release of interleukin and tumor necrosis factor, eventually altering cell function and promoting the occurrence and development of vascular diseases [17]. Based on these evidence, the expression levels of related factors in the serum of rats in each group were measured 14 days after a treatment: The serum levels of ET-1, ICAM-1, IL-6, and TNF-*α* in diabetic rats were increased, and the levels of NO and NOS were reduced, implying that the vascular endothelium of diabetic rats was damaged, leading to the release of inflammatory factors, affecting the wound healing. After treatment, the serum levels of ET-1, ICAM-1, IL-6, TNF-*α*, NO, and NOS exhibited no difference in rats treated with low-dose APS. The serum levels of ET-1, ICAM-1, IL-6, and TNF-*α* were reduced in rats treated with medium-dose APS, while the levels of NO and NOS were enhanced. The serum levels of ET-1, ICAM-1, IL-6, and TNF-*α* were further reduced in rats treated with high-dose APS, while the levels of NO and NOS were further enhanced. We observed that APS could increase the activity of NO and NOS and reduce ET-1 to protect vascular endothelium, in addition to inhibiting the release of inflammatory mediators, improving endothelial injury and maintaining the balance of vasomotor function (Figures 3(a)–3(f)).

The article "Astragalus Polysaccharides Promote Wound Healing in Diabetic Rats by Upregulating PETN and Inhibiting the mTOR Pathway" was retracted in 2023. Reasons: signs of a paper mill; compromised peer review; unreliable results or conclusions.

### 3.6. Expression of PTEN and mTOR Pathway-Related Proteins in Wound Tissues of Rats

There is evidence showing that APS-loaded fibrous mats can restore the microcirculation in or around skin wounds to expedite wound healing in diabetic rat models [4], indicating that APS has protective effects on the endothelium, but the mechanism has not yet been studied.

PTEN expression was detected by RT-qPCR, and the expression levels of PTEN and mTOR pathway-related proteins were determined by Western blot. PTEN mRNA and protein expression levels were reduced in the wound tissues of the diabetic rats at various time points, and the ratio of p-mTOR/mTOR protein was also significantly increased. PTEN expression in rats treated with high dose of APS was increased with time, on day 7 and day 14, and the p-mTOR/mTOR protein ratio was also decreased (Figures 4(a)–4(c)).

### 3.7. APS Improves the Healing of Diabetic Wounds by Upregulating PTEN and Inhibiting the mTOR Pathway

Next, we injected lentivirus knockdown vector (siRNA-PTEN) and lentivirus NC (siRNA-NC) locally into rats according to the grouping after intragastric administration within 3, 7, and 14 days after the skin wound. The rats were accordingly grouped into the model+siRNA-NC group, APS+siRNA-NC group, and APS+siRNA-PTEN group. The results showed that compared with the APS+siRNA-NC group, wound healing in the model+siRNA-PTEN group was improved, consistent with the above observation. Additionally, the results suggested that local injection of lentivirus knockdown vector siRNA-PTEN reversed the effects of APS. At 14 days after the wound establishment, rats injected with lentivirus knockdown vector siRNA-PTEN exhibited slow wound recovery; enhanced serum levels of ET-1, ICAM-1, IL-6, and TNF-*α*; reduced serum levels of NO and NOS; and decreased expression level of CD31, implying that siRNA-PTEN treatment damaged the blood vessel endothelium and released more inflammation mediators. The detection of PTEN and mTOR expression in rats by RT-qPCR and Western blot revealed that PTEN expression was inhibited and the phosphorylation level of mTOR was enhanced in rats injected with siRNA-PTEN (Figures 5(a)–5(i)).

The article "Astragalus Polysaccharides Promote Wound Healing in Diabetic Rats by Upregulating PETN and Inhibiting the mTOR Pathway" was retracted in 2023. Reasons: signs of a paper mill; compromised peer review; unreliable results or conclusions.

The aforementioned results indicate that APS could improve the healing of diabetic wounds by upregulating PTEN and inhibiting the mTOR pathway.

## 4. Discussion

Wound healing difficulties are a severe complication of diabetes, resulting in chronic wounds, prolonged hospitalization, and even limb amputation [18]. Physiological control of wound healing is an intricate process that depends on the interaction of many cells and mediators in a highly complicated temporal manner [19]. Although the mechanisms and specific functions in diabetic wound healing have been delineated to some extent, many basal pathophysiological processes remain unknown, and novel wound healing therapies are required to better comprehend this complex interplay. In this present study, we explored the possible mechanism of APS in treating diabetic wounds by observing the effects of APS on wound healing in diabetic rats and the involvement of PTEN and the mTOR pathway.

The action mechanism of APS for diabetes has been reported to focus on insulin secretion, insulin sensitivity, intestinal absorption of glucose, glucolipid metabolism in the liver, and regulation of gut microbiota, as well as antioxidant and anti-inflammatory activities [20]. Evidence has suggested that wound healing in diabetes is directly associated with poorly modulated serum glucose levels [21]. Firstly, STZ was injected into the tail vein of SD rats to induce a diabetic animal model, and an incision was made on the back to prepare a skin wound model. After successful modeling, the functions of APS on diabetic wound healing were explored, and findings suggested that APS could promote wound healing in diabetic rats. In line with our study, STZ-treated rats have been found to exhibit a reduction in body weight and plasma glucose, along with an improvement in insulin sensitivity upon treatment of APS [22]. Also, another research has implied that APS2-1 (a novel polysaccharide) had high potential in wound healing by suppressing inflammation, promoting cell cycle, and enhancing the secretion of repair factors [23]. Furthermore, it is reported that APS enhances the expression levels of proinflammatory cytokines (secretion of TNF-*α* and NO) in RAW264.7 cells [24]. All these data suggest that APS is significant in wound healing.

The article "Astragalus Polysaccharides Promote Wound Healing in Diabetic Rats by Upregulating PETN and Inhibiting the mTOR Pathway" was retracted in 2023. Reasons: signs of a paper mill; compromised peer review; unreliable results or conclusions.

The next step was to determine the possible mechanism of APS in treating diabetic wound healing. PTEN has been revealed to participate in some biological processes and impact angiogenesis via controlling endothelial cell biological functions [25]. A previous study showed that PTEN was able to successfully improve wound repair using electric signals [26]. A recent study also demonstrated that PTEN upregulation promoted wound repair *in vitro* and *in vivo* [13]. In our study, RT-qPCR and Western blot assay were implemented to observe the effects of APS on PTEN expression levels, and the findings suggested that APS inhibited PTEN expression in rats, which could effectively inhibit the promoting effect of APS on wound healing in diabetic rats. Similarly, PTEN inhibition has been implied to improve wound healing through changes in cellular mechanics [27]. As skin carcinogenesis remarkably elevates, mTOR inhibitors are considered as the first-line immunosuppression or more or less the first-line alternative in people who begin to develop skin cancer [28]. Squarize et al. disclosed that mTOR activation could induce cutaneous wound healing through the epithelial-specific suppression of PTEN, while pharmacological downregulation of mTOR delayed wound closure [29]. Based on these evidences, we speculated that APS might affect PTEN expression in diabetic rats, thereby affecting the mTOR pathway. With a series of experiments, we found that APS might be beneficial for wound healing in diabetic rats via the upregulation of PTEN and inhibition of the mTOR pathway. In similar studies, APS was shown to have a protective role by regulating mTOR expression [30]. Also, APS diminished the mTOR activity in pathological conditions and protected cells [5]. Furthermore, a recent research revealed that APS could decrease the phosphorylation of AKT together with mTOR (its downstream target protein) and upregulated PTEN expression, indicating that APS could block the activation of the I3K/AKT/mTOR pathway-associated proteins [31].

Despite the promising findings observed, there were some limitations that should be addressed. First, we only used rat models and whether these findings could be replicated in human models, such as human cell lines and organoids, is yet to be clarified. Second, it is widely known that type 1 diabetes is characterized by the autoimmune destruction of pancreatic *β* cells, and the association between APS treatment on pancreatic *β* cells and T cells, which might mediate diabetes and destroy insulin-producing *β* cells in the pancreatic islets, was not investigated. In addition, the functions of APS in patients with T2DM need to be further studied. Although there are many experimental studies on the effects and immunomodulation of APS, there is still a lack of clinical research. Further, insufficient studies on APS's structural characteristics also restrict its clinical research. Therefore, conducting more clinical research based on sufficient structural characterization studies in the future may be an important research direction.

The article "Astragalus Polysaccharides Promote Wound Healing in Diabetic Rats by Upregulating PETN and Inhibiting the mTOR Pathway" was retracted in 2023. Reasons: signs of a paper mill; compromised peer review; unreliable results or conclusions.

In conclusion, our study highlights that APS could promote wound healing in diabetic rats in a dose-dependent manner, and its mechanism might be related with the upregulation of PTEN and inhibition of the mTOR pathway, inhibition of inflammation, and regulation of vascular endothelial function. This study provides a theoretical basis and molecular mechanism for the treatment of refractory diabetic wounds.

## Figures and Tables

**Figure 1:** Basic condition and wound healing in rats. (a) The body weight change of rats in each group on the 0, 3^rd^, 7^th^, and 14^th^ days of skin wound establishment. (b) The blood glucose comparison of rats in each group on the 0, 3^rd^, 7^th^, and 14^th^ days of skin wound establishment. (c) Wound healing of rats at different time points in each group. (d) Comparison of wound healing rate of rats in each group. Data were expressed as mean ± SD, and comparisons among groups were determined by one-way analysis of variance. ^∗∗^*P* < 0.01 vs. the control group; ^#^*P* < 0.05 or ^##^*P* < 0.01 vs. the model group.

**Figure 2:** Histomorphology of rat wounds in each group. (a) H&E staining of granulation tissues in different groups at different time points (×200). (b) Masson staining of granulation tissues in different groups at different time points (×200). (c) Ki67 expression in each group was determined by IHC (×200). (d) CD31 immunohistochemical staining on granulation tissues (×200). (e) 14 days after modeling, the MVD was calculated. Data were expressed as mean ± SD, and comparisons among groups were determined by one-way analysis of variance. *N* = 6. ^∗∗^*P* < 0.01 vs. the control group; ^#^*P* < 0.05 or ^##^*P* < 0.01 vs. the model group.

**Figure 3:** Detection of expression of vascular endothelial-related factors and inflammatory factors in each group of rats. (a–c) Comparison of serum levels of vascular endothelial-related factors (ET-1, NO, and NOS) in rats. (d–f) Comparison of serum levels of inflammatory factors (ICAM-1, IL-6, and TNF-*α*) in rats. Data were expressed as mean ± SD, and comparisons among groups were determined by one-way analysis of variance. *N* = 6, three duplicate wells were set. ^∗∗^*P* < 0.01 vs. the control group; ^#^*P* < 0.05 or ^##^*P* < 0.01 vs. the model group.

The article "Astragalus Polysaccharides Promote Wound Healing in Diabetic Rats by Upregulating PETN and Inhibiting the mTOR Pathway" was retracted in 2023. Reasons: signs of a paper mill; compromised peer review; unreliable results or conclusions.

**Figure 4:** Expression of PTEN and mTOR pathway-related proteins in wound tissues of rats in each group. (a) RT-qPCR detection of PTEN mRNA expression level in wound tissues of rats in each group. (b) Western blot assay detection of PTEN protein expression in wound tissues of rats in each group. (c) Western blot assay detection of mTOR phosphorylation level in wound tissues of rats in each group. Data are expressed as mean ± SD, and comparisons among groups were determined by one-way analysis of variance. *N* = 6. ^∗∗^*P* < 0.01 vs. the control group; ^#^*P* < 0.05 or ^##^*P* < 0.01 vs. the model group.

**Figure 5:** APS inhibits the activation of the mTOR pathway by upregulating PTEN. (a–d) Comparison of serum levels of vascular endothelial-related factors (ET-1, NO, and NOS) in rats. (e) Comparison of serum levels of inflammatory factors (ICAM-1, IL-6, and TNF-*α*) in rats. (g) RT-qPCR detection of PTEN mRNA expression level in wound tissues of rats in each group. (h) Western blot assay detection of PTEN protein expression in wound tissues of rats in each group. (i) Western blot assay detection of mTOR phosphorylation level in wound tissues of rats in each group. Data are expressed as mean ± SD, and comparisons among groups were determined by one-way analysis of variance. *N* = 6. ^∗∗^*P* < 0.01 vs. the APS+siRNA-NC group.

## Data Availability

The data used to support the findings of this study are available from the corresponding author upon request.
